# Association between history of viral infections and melanoma mortality

**DOI:** 10.1016/j.heliyon.2024.e40353

**Published:** 2024-11-12

**Authors:** Nathan Shen, Polly Creveling, Joshua J. Horns, Josh Bleicher, John Hyngstrom, Tawnya Bowles, Michael Andreae, Tracy Onega, Elliot A. Asare

**Affiliations:** a Huntsman Cancer Institute, Salt Lake City, UT, 84112, USA; b University of Utah, Spencer Fox Eccles School of Medicine, Salt Lake City, UT, USA; c University of Utah Huntsman Cancer Institute, Department of Surgery, Salt Lake City, UT, USA; d Department of Surgery, Intermountain Medical Center, 5169 S Cottonwood Dr, Murray, UT, 84107, USA; e Department of Anesthesiology, University of Utah, Salt Lake City, UT, USA; f Department of Population Health Sciences, University of Utah, Salt Lake City, UT, USA

**Keywords:** Melanoma, VIs, Immune checkpoint inhibitors, PD-1

## Abstract

**Background:**

Viral infections (VIs) have been linked to T-cell exhaustion, a state that impacts the immune system's ability to mount an effective anti-tumor response. This immunosuppressive effect may potentially worsen outcomes in melanoma patients. This study investigates the relationship between a history of VIs and melanoma-specific mortality, with the goal of understanding whether prior history of Vis contribute to an increased risk of mortality in melanoma patients.

**Materials and methods:**

A retrospective review of patients in the Utah Population Database (1997–2020) was done. There were 17,754 eligible melanoma patients, with 2286 also having a history of viral infections. Multivariable Cox proportional hazard models were used to assess the effect of VI on melanoma-specific mortality.

**Results:**

History of VI was associated with a higher risk of melanoma-specific mortality (HR = 1.33, 95 % CI: 1.07–1.65, P = 0.01). No differences were observed in mortality among patients undergoing surgery and adjuvant immunotherapy.

**Conclusions:**

A history of viral infections was associated with higher melanoma-specific mortality. The mechanism of this association and relationship with different types of viral infections and duration of infections remain to be elucidated.

## 1 Introduction

Over the last decade, the US has observed a rise in the incidence rate of melanoma, but concurrently, a remarkable 30 % decrease in the mortality rate [[1], [2], [3]]. This reduction in fatalities can likely be attributed to the breakthroughs in innovative treatment modalities, including checkpoint inhibitors and targeted therapies [4].

Although immune checkpoint inhibitors have significantly reduced mortality for patients with unresectable stage III and IV melanoma [4,5], it remains unknown how the patient's unique immunologic milieu could be informative in predicting response to systemic therapy and estimating prognosis.

The prevalence of Viral infections (VIs) in the U.S. is a significant concern, with Hepatitis B and C (HBV and HCV) estimated to affect 3.5 million (2.5–4.7 million) and 850,000 (730,000–2.2 million) individuals respectively [6]. Over 50 % of people living with hepatitis do not know they have the condition [7,8]. The prevalence of Human Immunodeficiency Virus (HIV) in the US is estimated at 1.2 million, with 13 % not knowing they are infected [9,10]. In many cases of viral infections (VIs), lasting antigen exposure is able to upregulate PD-1, promoting T-cell exhaustion, immune tolerance, and NK cell compromise [11,12]. Some studies have reported worse outcomes for patients with various cancer types, including melanoma, who had increased expression of PD-1 or PD-L1 checkpoint mediators [13,14]. Based on knowledge of the effect of infection on T cell function, it is hypothesized that melanoma patients with history of VIs will have increased mortality due to immune dysregulation.

Our key objective is to investigate the relationship between a history of VIs and melanoma specific mortality in a unique population database from a region of the US with high incidence of melanoma. Unveiling this relationship could allow for better screening and treatment strategies for certain high-risk populations.

## 2 Methods

We utilized a subgroup of patients in the Utah Population Database (UPDB) diagnosed with melanoma from 1997 to 2020. 10.13039/100007747The University of Utah Institutional Review Board (IRB) granted an exemption for this study (IRB# 00129,538). The UPDB is a comprehensive population database, that links to the Utah Cancer Registry which captures data of all cancer diagnoses and treatment within the state of Utah. For this study, only patients who received their healthcare through the University of Utah Health systems were included (defined as at least two outpatient visits within the University of Utah Health system).

### 2.1 The effect of VI on melanoma specific mortality

We identified all melanoma cases in Utah between 1997 and 2020. For each melanoma patient we recorded their first diagnosis of melanoma, their first and last year in Utah, birth date, their date and cause of death, race/ethnicity, history of any other type of cancer, and average elevation of residency. For each patient we also recorded their first diagnosis of VI (if any). VI was defined as a documented history in medical records of Hepatitis B virus (HBV), Hepatitis C virus (HCV), Human immunodeficiency virus (HIV), Cytomegalovirus (CMV), Human T-lymphotropic virus (HTLV), Human papilloma virus (HPV), Herpes simplex virus (HSV), Epstein-Barr virus (EBV), or VI not otherwise specified. The duration of viral infection is unknown for our subgroups and therefore we were unable to distinguish between acute and chronic infections. Patients were excluded if they left Utah prior to 1997 (when diagnostic records became available), if we lacked information on when they first entered Utah, or if they had a diagnosis of VI or melanoma prior to their first residence in Utah.

To assess how VI impacted mortality in melanoma patients, we ran a Cox proportional hazard model (CPH). VI was our primary predictor of interest. We also controlled for sex, race/ethnicity (defined as non-Hispanic White or other), and average elevation of residence. Patients were followed from their initial melanoma diagnosis until melanoma-specific mortality. Patients were censored when they left the state.

To assess differences in treatment efficacy for melanoma patients with VI, we found all patients undergoing surgery and receiving adjuvant therapy. We ran two additional CPH models in this subgroup looking at time from initial melanoma diagnosis to melanoma-specific mortality. Covariates and censoring were as described above. Statistical analysis was performed using R (version 4.3).

## 3 Results

We identified 212,508 patients with a melanoma diagnosis in the UPDB, of whom 17,754 met the inclusion criteria for analysis.

The median age at melanoma diagnosis was 62 [IQR = 49–72] (Table 1). Utah's population predominantly identifies as white and 17,304 (97.5 %) of melanoma patients were white. The average elevation at residence was 4549 feet [4390–4786]. Among all patients with melanoma, 10,140 (57.1 %) were male. Most patients were born in the 1940s and 1950s (22.1 % and 22.0 % respectively). Two thousand two hundred and seventy-six (12.8 %) melanoma patients were also diagnosed with VI.

**Table 1:** Demographic data of eligible patients with melanoma from the Utah population database (1997–2020).

Variable	Melanoma Patients
Total	17,754 (100 %)

Median age, IQR	62 (49–72)

Sex	

Male	10,140 (57.11 %)
Female	7614 (42.89 %)

Birth decade	

pre-1900	0 (0.00 %)
1900	13 (0.07 %)
1910	264 (1.49 %)
1920	1492 (8.40 %)
1930	2945 (16.59 %)
1940	3923 (22.10 %)
1950	3905 (22.00 %)
1960	2398 (13.51 %)
1970	1692 (9.53 %)
1980	938 (5.28 %)
1990	181 (1.02 %)
2000	3 (0.02 %)

NIH race	

American Indian/AK Native	10 (0.06 %)
Asian	21 (0.12 %)
HI/PI	9 (0.05 %)
Black/African American	7 (0.04 %)
White	17,304 (97.47 %)
Multiple	328 (1.85 %)
Unknown	75 (0.42 %)

Ethnicity	

Latino	2590 (14.59 %)
Non-Latino	15,050 (84.77 %)
Unknown	114 (0.64 %)

Education	

Some high school or less	933 (5.26 %)
High school degree	3151 (17.75 %)
Some college	4107 (23.13 %)
College degree	2622 (14.77 %)
Post-college	2815 (15.86 %)
Unknown	4126 (23.24 %)

Elevation	4548.7 (4390.1–4786)

Key: AK: Alaskan Native, HI/PI: Hawaiian/Pacific Islander.

Less than 15 % of the subgroup experienced melanoma specific mortality. Presence of viral infection was associated with a 33 % increased risk of melanoma specific mortality in our subgroup (HR = 1.33, 95 % CI: 1.07–1.65 [P = 0.01]) [Table 2] [Fig. 1]. No statistically significant associations were found between viral infections and melanoma incidence and recurrence.

**Table 2:** Results of Multivariable analysis of factors associated with melanoma-specific mortality.

Factors	Hazard Ratio (HR)	95 % Confidence Interval (CI)	p-value
VI	1.33	1.07–1.65	0.01
Elevation	0.91	0.86–0.97	0.003
Sex (male)	1.71	1.48–1.97	0.00
Race/Ethnicity (Non-Hispanic White)	1.14	0.94–1.34	0.21

**Key:** Effect of viral infection (VI) relative to non-VI, effect of elevation represents increase of 500 feet, effect of sex relative to female, effect of race relative to Hispanic or non-White.

**Fig. 1:** Melanoma-specific mortality in matched subgroups with and without viral Infection. Key: Blue: patients without viral infection; Red: patients with viral infection. Follow-up truncated at 20 years for clarity of presentation.

Of the 1238 patients who underwent surgery and received adjuvant immunotherapy (n = 1174 for non-viral infection subgroup and n = 64 for viral infection subgroup). Over the course of the follow-up for this small subgroup, there was no statistically significant difference in melanoma-specific mortality between the group with viral infection and melanoma and those with melanoma alone (HR 1.35,95 % CI: 0.97–1.88 [P = 0.99]; HR 1.29, 95 % CI: 0.68–2.33 [P = 0.46]) [Table 3] [Fig. 2].

**Table 3:** Results of Multivariable Analysis of Factors Associated with Overall Mortality and Melanoma Specific Mortality in patients receiving surgery and adjuvant immunotherapy.

Factors	HR for Overall Mortality (95 % CI; p-value)	HR for Melanoma-Specific Mortality (95 % CI; p-value)
VI	1.35 (0.97–1.88; p = 0.08)	1.26 (0.68–2.33; p = 0.46)
Elevation	0.94 (0.85–1.04; p = 0.23)	0.95 (0.79–1.15; p = 0.60)
Sex (male)	1.39 (1.08–1.78; p = 0.01)	1.49 (0.96–2.32; p = 0.07)
Race/Ethnicity (Non-Hispanic White)	0.80 (0.60–1.07; p = 0.129)	0.74 (0.44–1.24; p = 0.25)

**Key:** Model outputs for overall mortality (left), and melanoma-specific mortality (right) in patients undergoing immunotherapy and surgery. Effect of viral infection (VI) relative to non-VI, effect of elevation represents increase of 500 feet, effect of sex relative to female, effect of race relative to Hispanic or non-White.

**Fig. 2:** Melanoma recurrence-free survival and mortality for subgroups who received surgery and adjuvant immunotherapy.

## 4 Discussion

Our study using the UPDB demonstrated that a history of VIs increased the risk of melanoma-specific mortality in the subgroup of patients with viral infection and melanoma compared to those with melanoma alone. To our knowledge, this is the largest retrospective study using a unique comprehensive population database to assess the effect of a history of VIs on melanoma specific mortality. Our research adds to the growing body of literature investigating the impact of immunosuppressive states on melanoma mortality.

We found increased mortality in patients with VI and melanoma compared to melanoma alone. This adverse effect may be due to several mechanisms such as immunosuppression, inflammatory responses, and direct viral interactions with melanoma cells and the modulation of the tumor microenvironment. For example, several studies have documented how chronic viral infections promote CD8^+^ T-cell exhaustion via increased expression of the PD-1/PD-L1 pathway [15,16]. Specifically, high levels of circulating soluble PD-L1 have been linked to poor prognosis. They can serve as a prognostic biomarker in melanoma and other cancers [[17], [18], [19]], as they may bind to PD-1 on T-cells, reinforcing immune suppression and exhaustion. Our findings provide support to these observations, suggesting that VIs may upregulate PD-1 expression and potentiate immune dysfunction, contributing to increased MSM. However, further studies are needed to elucidate the precise biological pathways governing this definitively observed increased in MSM, as the severity, duration, and specific type of viral infection may differentially affect these mechanisms. Within the subset of patients treated with surgical intervention followed by adjuvant immunotherapy, no statistically significant association was found between viral infections and the recurrence of melanoma, nor with overall or disease-specific mortality. This finding may be limited by our relatively small sample size, particularly among participants afflicted with both viral infection and melanoma. Patients with viral infections such as HIV, have frequently been reported to experience higher rates of cancer-specific mortality across a broad spectrum of cancers, including colorectal, lung, melanoma, and breast cancers [20]. In this retrospective population database, we did not have data on duration of viral infections, reactivation of infections and concomitant immunosuppressive factors which may influence these associations with risks of melanoma, recurrence, and mortality.

Our study has a few important limitations that merit discussion. Firstly, while the UPDB allows for analysis with a substantial sample size, it largely represents the predominantly white population in Utah. This factor may restrict the generalizability of our findings to a more racially diverse demographics. Secondly, our dataset did not permit stratification based on distinct types of VIs, the duration or severity of VIs, lifestyle factors, sun exposure habits, VI treatment, and other immunosuppressive states. Also, our subgroup spanned American Joint Committee on Cancer (AJCC) Staging System 4th, 5th, 6th, 7th and 8th editions and this prevented us from stratifying by stage as we did not have the data elements to convert the old stages to contemporary AJCC stage. Furthermore, because VI is often diagnosed in an outpatient setting, it is possible that some of the people we identified as non-VI controls were diagnosed in another setting. Additionally, we would like to acknowledge that our reliance on zip code data for geographical analysis may not account for the full residential history of patients such as the duration they have lived at their current elevation or their childhood exposure. Lastly, the retrospective nature of our study leaves room for potential unmeasured confounders that could affect the interpretation of our findings such as surveillance bias. These highlighted limitations underscore the need for further prospective research to validate and expand upon our findings.

## 5 Conclusion

Our retrospective analysis of a population database revealed an associated increased risk of melanoma-specific mortality in subgroups with viral infections and melanoma, compared to those with melanoma alone. Data on specific types of viral infections, duration of infection, and concomitant immunosuppressive states are needed to elucidate this important relationship for populations who have melanoma or are at risk for melanoma.

## CRediT authorship contribution statement

**Nathan Shen:** Writing – review & editing, Writing – original draft, Conceptualization. **Polly Creveling:** Writing – review & editing, Writing – original draft. **Joshua J. Horns:** Visualization, Formal analysis, Data curation. **Josh Bleicher:** Writing – review & editing. **John Hyngstrom:** Writing – review & editing. **Tawnya Bowles:** Writing – review & editing. **Michael Andreae:** Writing – review & editing. **Tracy Onega:** Data curation. **Elliot A. Asare:** Writing – review & editing, Writing – original draft, Visualization, Validation, Supervision, Resources, Project administration, Methodology, Investigation, Funding acquisition, Formal analysis, Data curation, Conceptualization.

## Data availability

The data for this study were obtained from the Utah Population Database (UPDB). There are restrictions to the availability of this data, which is used under license for this study. Data can be accessed with permission from the Utah Population Database (UPDB).

## Declaration of competing interest

The authors declare no conflicts of interest regarding the publication of this manuscript.
